The article "Prognostic value of magnetic resonance imaging features in low-grade gliomas" was published in 2019. Journal: Biosci Rep.

# Prognostic value of magnetic resonance imaging features in low-grade gliomas

**DOI:** 10.1042/BSR20190544

**Published:** 2019-06-04

**Authors:** Liang Deng, Liangfang Shen, Lin Shen, Zhao Zhao, Yingpeng Peng, Hongjiao Liu, Haipeng Liu, Guangying Zhang, Zhanzhan Li, Kai Li, Erdong Shen, Yuanyuan Liu, Chao Liu, Xinqiong Huang

**Affiliations:** 1 Department of Oncology, Xiangya Hospital, Central South University, Changsha, China; 2 Department of Head and Neck Oncology, The Cancer Center of the Fifth Affiliated Hospital Sun Yat-Sen University, Zhuhai, China; 3 Department of Oncology, No.1 Traditional Chinese Medicine Hospital in Changde, Changde, China; 4 Department of Radiology, Xiangya Hospital, Central South University, Changsha, China; 5 Department of Oncology, Yueyang First People’s Hospital, Yueyang, China; 6 Department of Human Resources, Xiangya Hospital, Central South University, Changsha, China; 7 Department of Epidemiology and Health Statistics, Xiangya School of Public Health, Central South University, Changsha, China

**Keywords:** Cyst, Low-grade glioma, Magnetic Resonance Imaging, Necrosis, Prognosis, Ring-like enhancement

## Abstract

**Introduction:** The treatment strategy for low-grade gliomas (LGGs) is still controversial, and there are no standardized criteria to predict the prognosis of patients with LGGs. Magnetic resonance imaging (MRI) is a routine test for preoperative diagnosis for LGG and can reflect the destructive features for the tumor. In the present study, we aimed to explore the relationship between the MRI features and prognosis in patients with LGG.

**Methods:** Clinical data of 80 patients with pathologically proved LGGs between January 2010 and December 2016 were analyzed retrospectively. MRI features were classified as contrast enhancement pattern (focal enhancement, diffuse enhancement and ring-like enhancement), necrosis and cysts based on the preoperative MR images. Kaplan–Meier method and multivariate analysis were performed on the data by SPSS software to explore the prognostic significance of MRI features.

**Results:** Patients with cystic LGG had a significantly longer 5-year progression-free survival (PFS) than that with no cyst (90.9 ± 8.7 vs 65.7 ± 9.1%, *P*=0.045). Multivariate analysis further verified cyst as an independent prognosis factor for PFS (*P*=0.027, hazard ratio [HR] = 0.084). Additionally, patients with ring-like enhancement exhibited significantly longer 5-year PFS time in the Kaplan–Meier survival curves (100 vs 67.2 ± 7.7%, *P*=0.049). There was no significant difference in PFS and overall survival (OS) between patients with or without necrosis.

**Conclusion:** Our study suggests that cyst formation and ring-like enhancement on preoperative MR images can be useful to predict a favorable prognosis in patients with LGGs.

## Introduction

Low-grade gliomas (LGGs) are primary brain tumors that arise from the glial cells of the central nervous system [1,2]. LGGs are constituting approximately 30% of gliomas, and the morbidity age is younger than high-grade gliomas. LGGs are classified into grade I and grade II by the World Health Organization (WHO), which are well-differentiated [3]. However, the features of WHO grade II tumors and WHO grade I tumors are very different, not only in terms of histopathologic features but also in the clinical prognosis [4,5]. WHO grade I gliomas are benign tumors that can be cured by radical surgery. Instead, WHO grade II gliomas have a certain rate of recurrence and increase in grade with the passage of time [6,4,7]. The most common LGGs are the WHO grade II gliomas, and include astrocytomas, oligodendrogliomas, and mixed oligoastrocytomas [8,9].

The data of EORTC study 22844 has verified some unfavorable prognostic factors influencing survival for LGGs, including age ≥40, astrocytoma, the maximum diameter of tumor ≥6 cm, tumor crosses midline, and preoperative neurological impairment [10]. Furthermore, combined loss of 1p and 19q is independent prognosis factor of prolonged survival in LGG patient which originated from oligodendrocytes [11]. IDH mutation was also found to be related to the prognosis of LGGs [12]. However, in addition to the above-mentioned factors, we found some magnetic resonance imaging (MRI) features of the tumor which might influence the prognosis of LGG patients in the clinical work, but it has rarely been studied so far. Therefore, take the imaging features into account could strengthen the predicting system for prognosis in patients with LGGs.

In terms of China’s current economic and medical situation, many grass-root hospitals were unable to develop the genetic testing and multi-functional MRI because many patients’ families cannot afford the costs for the above inspections. Instead, most hospitals develop regular MRI which is comparatively cheap and can confirm the lesion morphologically. Hence in the present study, we focused on the features of the regular MRI to explore its prognostic significance. If we can take full advantage of regular MRI to estimate prognosis and guide treatment, it will benefit patients in developing countries in Africa, Asia and Latin America.

In the clinic, MRI is a routine test for the preoperative diagnosis of glioma. Several studies showed that contrast enhancement was significantly related with the prognosis of patients with gliomas. The integrated analysis of Gutman et al. [13] showed that the proportion of contrast enhancement of tumor possibly suggests poor survival in patients with glioblastomas. Previous researches have highlighted that tumor necrosis is correlated with a poor prognosis in malignant glioma [14,15]. Additionally, Kaur et al. [16] demonstrated that the presence of a cyst in tumor does not significantly affect overall survival (OS) in patients with glioblastomas. Another study showed that presence of intramedullary cysts significantly improved progression-free survival (PFS) in patients with low-grade astrocytomas of the spinal cord [17]. Nevertheless, the number of studies concentrating on the prognostic significance of preoperative MRI features in LGGs are limited. In the present study, we aimed to fill the gap of knowledge by exploring the relationship between the MRI features and survival outcome, and therefore to find a more reasonable forecast method for the prognosis of patients with LGGs.

## Methods

### Patients

The clinical and radiologic data of 80 patients with pathologically proved LGGs (WHO grade II) between January 2010 and December 2016 were analyzed retrospectively. All patients received radiotherapy plus chemotherapy at Xiangya Hospital of Central South University (Changsha, China), they were followed until December 2017. The medium follow-up period was 34.5 (range: 1–83) months. Patients who died of non-glioma-based causes were excluded from the study sample. Preoperative MRI scans of all patients were consulted and none of these had previous diagnosis of any other brain tumor in the past. All patients received concurrent chemoradiotherapy. The prescribed radiotherapy doses for intensity-modulated radiation therapy (IMRT) were 44–60 Gy, the medium dose was 50.68 Gy. All patients received chemotherapy as temozolomide (TMZ) (50 mg*7s, Tasly Holding Group Co. Ltd., China) after operation, consisting 75 mg/m^2^ per day. Clinical variables from patients included age, gender, tumor morphology, tumor residual, preoperative neurological impairment and histopathology. The median age of onset was 36 years (range, 9–68 years). The preoperative KPS of these patients was 80 (range, 30–90). Table 1 summarized the clinical characteristics of these patients with LGG. The present study was approved by the Ethics Committee in Xiangya Hospital of Central South University.

**Table 1:** Variables associated with PFS and OS in the entire cohort (*n*=80)

Characteristics	Total cases	Progression	Progression free	*P* value	Death	Survival	*P* value
Enhancement							
Total of contrast enhancement	48.75% (39)	10.00% (8)	38.75% (31)	0.270	7.50% (6)	41.25% (33)	0.496
Focal enhancement	23.75% (19)	7.50% (6)	16.25% (13)		5.00% (4)	18.75% (15)	
Diffuse enhancement	12.50% (10)	2.50% (2)	10.00% (8)		2.50% (2)	10.00% (8)	
Ring-like enhancement	12.50% (10)	0.00% (0)	12.50% (10)		0.00% (0)	12.50% (10)	
Non-contrast enhancement	51.25% (41)	12.50% (10)	38.75% (31)		8.75% (7)	42.50% (34)	
Ring-like enhancement							
Yes	12.50% (10)	0.00% (0)	12.50% (10)	0.069	0.00% (0)	12.50% (10)	0.136
No	87.50% (70)	22.50% (18)	65.00% (52)		16.25% (13)	71.25% (57)	
Necrosis							
Yes	18.75% (15)	5.00% (4)	13.75% (11)	0.668	3.75% (3)	15.00% (12)	0.662
No	81.25% (65)	17.50% (14)	63.75% (51)		12.50% (10)	68.75% (55)	
Cyst							
Yes	17.50% (14)	1.25% (1)	16.25% (13)	0.130	1.25% (1)	16.25% (13)	0.309
No	82.50% (66)	21.25% (17)	61.25% (49)		15.00% (12)	67.50% (54)	
Age							
≥40	42.50% (34)	10.00% (8)	32.50% (26)	0.850	8.75% (7)	33.75% (27)	0.366
<40	57.50% (46)	12.50% (10)	45.00% (36)		7.50% (6)	50.00% (40)	
Gender							
Male	55.00% (44)	10.00% (8)	45.00% (36)	0.307	10.00% (8)	45.00% (36)	0.605
Female	45.00% (36)	12.50% (10)	32.50% (26)		6.25% (5)	38.75% (31)	
KPS							
≥70	91.25% (73)	21.25% (17)	70.00% (56)	0.586	16.25% (13)	75.00% (60)	0.222
<70	8.25% (7)	1.25% (1)	7.50% (6)		0.00% (0)	8.75% (7)	
Diameter							
≥6 cm	53.75% (43)	20.00% (16)	33.75% (27)	0.001	15.00% (12)	38.75% (31)	0.002
<6 cm	46.25% (37)	2.50% (2)	43.75% (35)		1.25% (1)	45.00% (36)	
Tumor cross midline							
Yes	33.75% (27)	11.25% (9)	22.50% (18)	0.099	6.25% (5)	27.50% (22)	0.695
No	66.25% (53)	11.25% (9)	55.00% (44)		10.00% (8)	56.25% (45)	
Tumor residual							
Yes	57.50% (46)	12.50% (10)	45.00% (36)	0.850	8.75% (7)	48.75% (39)	0.771
No	42.50% (34)	10.00% (8)	32.50% (26)		7.50% (6)	35.00% (28)	
Preoperative neurological impairment							
Yes	70.00% (56)	16.3% (13)	53.8% (43)	0.055	13.8% (11)	56.3% (45)	0.209
No	30.00% (24)	6.3% (5)	23.8% (19)		2.5% (2)	27.5 (22)	
Histopathology							
Astrocytoma histology subtype	80.00% (64)	21.25% (17)	58.75% (47)	0.082	15.0% (12)	65.0% (52)	0.225
Non-astrocytoma histology subtype	20.00% (16)	1.25% (1)	18.75% (15)		1.3% (1)	18.8% (15)	

### Classification of MRI features

All patients received pre-surgical MRI scans using the 1.5-T Siemens Vision Plus scanner (Erlangen, Germany). The sequences contained T1-weighted imaging (T1-W), T2-weighted imaging (T2-W), and contrast-enhanced T1-W. We measured the unidimensional maximum diameter on the T2-W images [18]. To determine the residual tumor after operation, preoperative MRI scans and MR images within 3 days after operation were compared on tissue volumes [18]. Enhancement which was defined as partial regions of the tumor showed a significant increase in the signal intensity on contrast-enhanced T1-W images [19,20] (Figure 1). The signal intensity from the marked enhanced area can be close to that of fat. Depending upon the morphology of the largest enhanced region in the tumor, the patterns of enhancement were divided into three categories: focal enhancement, diffuse enhancement and ring-like enhancement. The focal enhancement pattern was defined as a well-defined enhancing area with a relatively smooth border [20] (Figure 1B). In contrast, the diffuse enhancement pattern was defined as a not well-defined enhancing area with rough border [20] (Figure 1C). The ring-like enhancement pattern was defined as a cystic necrosis surrounding by a contrast-enhanced border [19,20] (Figure 1D). Necrosis was defined as a region that exhibited high-intensity T2-W signals, but low intensity on T1W signals, and with an irregular border [21] (Figure 1E). Cyst was a well-defined and rounded region which had an extremely high signal intensity on T2-W images but a low signal on T1-W images, with a thin, regular and smooth wall [15] (Figure 1F). According to the above classification methods, the MR images of tumor were assessed in a blinded fashion by two senior radiologists.

**Figure 1:** Representative images of classification of contrast enhancement patterns T2-W images (the first line) and contrast-enhanced T1-W images (the second and bottom lines) of different MRI features were exhibited in LGGs. (**A**) Non-enhanced pattern; (**B**) Focal enhancement pattern; (**C**) Diffuse enhancement pattern; (**D**) Ring-like enhancement pattern; (**E**) Necrosis; (**F**) Cysts.

### Statistical analysis

All the data collected from the study were analyzed by SPSS version 23.0 (IBM Corp, Armonk, NY, U.S.A.). We used the chi-squared tests to determine the distribution of clinical characteristics of all patients with LGGs and compare the differences between each variable which is associated with PFS or OS. Survival curves were calculated by using the Kaplan–Meier method to compare the PFS and OS between patient cohorts, and differences were tested by the log-rank test. The Cox proportional hazards model was used to identify the independent prognosis indicator in the multivariate analysis. *P*≤0.05 suggests a statistically significant difference and all tests were two-sided.

## Results

### Patients’ clinical characteristics

A total of 80 patients with LGG (WHO grade II) were included in this retrospective study. In the cohort, 34 (42.5%) patients were 40 years or older and 46 (57.5%) patients were younger than 40. Forty-four (55%) patients were male and 36 (45%) patients were female. The preoperative KPS of 73 (91.25%) patients was greater than or equal to 70, 7 (8.25%) patients were less than 70. According to the preoperative MR images, the tumor of 27 (33.75%) patients crossed the brain midline and extended into another side of the brain hemispheres, the growth of tumor in 53 (66.25%) patients was limited to the one side of the brain hemisphere. By comparing the preoperative and post-operative MR images, 46 (57.5%) patients had the tumor residual after the surgery, 34 (42.5%) patients had no tumor residual. Preoperatively, 56 (70.0%) patients have appeared neurologic deficit, other 24 (30.0%) patients were not. Among all 80 patients, 64 (80%) were pathologically diagnosed with astrocytic component, and 16 (20%) with oligodendrogliomas. No significant differences in PFS or OS were observed between different groups with above-mentioned clinical variables (Table 1). In contrast, there were significant differences among patients with different tumor size in PFS (*P*=0.001) and OS (*P*=0.002). The diameter of 43 (53.8%) patients was bigger or equal to 6 cm and of 37 (46.3%) patients was smaller than 6 cm.

### Imaging features

Among all patients, 39 (48.8%) tumors demonstrated T1 contrast enhancement. Furthermore, the tumor contrast enhancement included three patterns: 19 (23.8%) cases with focal enhancement, 10 (12.5%) cases with diffuse enhancement, and 10 (12.5%) with ring-like enhancement. There was no statistical significance in PFS and OS between these enhancement pattern and non-contrast enhancement group. Significantly, of those with ring-like enhancement tumor, no one experienced tumor recurrence or disease progression. Therefore, we divided all patients into two groups for further study: tumor with and without ring-like enhancement. Tumor residual after surgery was significantly different between the patients with ring-like enhancement tumor and those without ring-like enhancement tumor (*P*=0.026, *P*=0.011; Table 2a). The ratios of necrosis and cyst among patients with LGGs were compared. The tumor of 15 (18.8%) patients had necrosis, of 65 (81.2%) patients with no necrosis, and the difference of clinical variables were explored in tumors with or without necrosis was not statistically significant (Table 2b). It seems that tumors with astrocytoma histology were more prone to have cyst. We found that 14 (17.6%) patients had cysts. The histopathology of these tumors with cysts were all astrocytoma histology subtype, the difference of which was statistical significant (*P*=0.039; Table 2c).

**Table 2a:** Clinical characteristics of all patients with LGGs

Characteristics	Ring-like enhancement		*P*-value
	Y	N	
Age (≥40/<40)	6/4 (7.5%/5.0%)	28/42 (35.0%/52.5%)	0.231
Gender (male/female)	7/3 (8.8%/3.8%)	37/33 (46.3%/41.3%)	0.308
KPS (≥70/<70)	8/2 (10.0%/2.5%)	65/5 (81.3%/6.3%)	0.178
Diameter (≥6 cm/<6 cm)	7/3 (8.8%/3.8%)	36/34 (45.0%/42.5%)	0.271
Tumor cross midline (Y/N)	5/5 (6.3%/6.3%)	22/48 (27.5%/60.0%)	0.245
Tumor residual (Y/N)	9/1 (11.3%/1.3%)	37/33 (46.3%/41.3%)	0.026
Preoperative neurological impairment (Y/N)	7/3 (8.8%/3.8%)	49/21 (61.3%/26.3%)	0.630
Histopathology (astro-/non-astro)	9/1 (11.3%/1.3%)	55/15 (68.8%/18.8%)	0.398

**Table 2b:** Clinical characteristics of all patients with LGGs

Characteristics	Necrosis		*P* value
	Y	N	
Age (≥40/<40)	8/7 (10.0%/8.8%)	26/39 (32.5%%/48.8%)	0.346
Gender (male/female)	9/6 (11.3%/7.5%)	35/30 (43.8%/37.5%)	0.666
KPS (≥70/<70)	14/1 (17.5%/1.3%)	59/6 (73.8%/7.5%)	0.751
Diameter (≥6 cm/<6 cm)	10/5 (12.5%/6.3%)	33/32 (41.3%/40.0%)	0.266
Tumor cross midline (Y/N)	8/7 (10.0%/8.8%)	19/46 (23.8%/57.5%)	0.075
Tumor residual (Y/N)	10/5 (12.5%/6.3%)	36/29 (45.0%/36.3%)	0.426
Preoperative neurological impairment (Y/N)	9/6 (11.3%/7.5%)	47/18 (58.8%/22.5%)	0.348
Histopathology (astro-/non-astro)	11/4 (13.8%/5.0%)	53/12 (66.3%/15.0%)	0.474

**Table 2c:** Clinical characteristics of all patients with LGGs

Characteristics	Cyst		p value
	Y	N	
Age (≥40/<40)	7/7 (8.4%/8.8%)	27/39 (33.8%/48.8%)	0.532
Gender (Male/Female)	5/9 (6.3%/11.3%)	39/27 (48.8%/33.8%)	0.110
KPS (≥70/<70)	11/3 (13.8%/3.8%)	62/4 (77.5%/5.0%)	0.065
Diameter (≥6 cm/<6 cm)	9/5 (11.3%/6.3%)	34/32 (42.5%/40.0%)	0.384
Tumor cross midline (Y/N)	4/10 (5.0%/12.5%)	23/43 (28.7%/53.8%)	0.652
Tumor residual (Y/N)	8/6 (10.0%/7.5%)	38/28 (47.5%/35.0%)	0.976
Preoperative neurological impairment (Y/N)	10/4 (12.5%/5.0%)	46/20 (57.5%/25.0%)	0.898
Histopathology (Astro-/Non-astro)	14/0 (17.5%/0.0%)	50/16 (62.5%/20.0%)	0.039

### Association of MRI with survival

We used the Kaplan–Meier survival curves and log-rank test to explore the association between each MRI feature with PFS and OS. As we can see from the survival curve (Figure 2A), patients with a ring-like enhancing tumor had a significantly longer 5-year PFS than those with no contrast-enhancing tumor or other patterns of enhancing tumor (100 vs 67.2 ± 7.7%, *P*=0.049; Table 3). Kaplan–Meier analysis also showed that cysts were significantly associated with PFS (*P*=0.045; Figure 2E). Patients with cystic tumor exhibited longer 5-year PFS (90.9 ± 8.7 vs 65.7 ± 9.1%, *P*=0.045; Table 3). Nevertheless, ring-like enhancement and cysts did not reach statistical significance for OS (Figure 2B,F and Table 3). In addition, presence of necrosis was not significantly associated with the prognosis in LGGs (Figure 2C,D). Multivariate analysis (Table 4) indicated that cysts [*P*=0.027; hazard ratio (HR), 0.084] and the diameter of tumor (*P*=0.002; HR, 12.123) were independent prognostic factors for PFS in patients with LGGs. Additionally, multivariate Cox regression analysis demonstrated that the diameter of tumor was significantly associated with OS (*P*=0.006; HR, 20.057).

**Figure 2:** Kaplan–Meier curves of progression-free survival and overall survival Correlations between (**A,B**) ring-like enhancement, (**C,D**) necrosis, (**E,F**) cyst and PFS and OS in the entire cohort.

**Table 3:** MRI features as prognostic factors for PFS and OS

Characteristics	Number of patients	Survival			
		5-year PFS	*P*-value	5-year OS	*P*-value
All patients	80	76.6 ± 5.5%		81.5 ± 4.9%	
Ring-like enhancement					
Yes	10	100%	0.049	100%	0.113
No	70	67.2 ± 7.7%		78.2 ± 5.7%	
Necrosis					
Yes	15	36.9 ± 27%	0.705	43.1 ± 30.8%	0.842
No	65	62.9 ± 10.2%		80.2 ± 5.7%	
Cyst					
Yes	14	90.9 ± 8.7%	0.045	90.0 ± 9.5%	0.211
No	66	65.7 ± 9.1%		68.2 ± 11.6%	

**Table 4:** Statistically significant prognosis indicators evaluated by multivariate analysis in the entire cohort

Characteristics	PFS			OS		
	*P*-value	HR	95%CI	*P*-value	HR	95%CI
Cyst (Y/N)	0.027	0.084	0.009–0.755	0.129	0.191	0.022–1.617
Age (≥40/<40)	0.867	1.099	0.363–3.332	0.550	1.475	0.412–5.275
Gender (male/female)	0.502	0.687	0.230–2.053	0.643	1.375	0.358–5.275
Diameter (≥6 cm/<6 cm)	0.002	12.133	2.441–60.299	0.006	20.057	2.363–170.269
Tumor cross midline (Y/N)	0.908	0.927	0.255–3.367	0.929	0.938	0.229–3.843
Residual (Y/N)	0.232	0.528	0.185–1.505	0.105	0.357	0.103–1.238
KPS (≥70/<70)	0.231	3.754	0.431–32.709	0.983	2.432	0.597–32.715
Preoperative neurological impairment (Y/N)	0.502	2.709	0.751–9.773	0.074	4.663	0.861–25.237
Histopathology (astro-/non-astro)	0.102	5.898	0.703–49.515	0.347	2.913	0.314–27.001

## Discussion

In this retrospective study, we explored the significance of preoperative MRI features in predicting the prognosis of patients with LGGs (WHO grade II). In the clinical work, MRI is an important routine method for the preoperative diagnosis of gliomas and evaluation of their treatment response. Our study analyzed several MRI features and found that cyst formation on preoperative MR images was an independent favorable prognostic factor for LGGs. In addition, our study suggested that ring-like enhancement pattern was associated with better prognosis in patients with LGGs.

Several studies have reported that the enhancement pattern of tumor can affect the prognosis of patients with high-grade gliomas. A previous study found that contrast enhancement was associated with poor prognosis and decreased survival in patients with anaplastic astrocytomas [22]. In addition, the study pointed that heterogeneously enhancing tumors appear to have poorer outcomes when compared with ring-like enhancing and nodular enhancing tumors. Previous studies have shown that enhancement on preoperative MR images was an independent adverse factor for prognosis in glioblastoma [14,23]. However, another retrospective study found the enhancement was not significantly related with OS of patients with glioblastoma and anaplastic glioma on multivariate analysis [21]. Therefore, we can see that the prognostic significance of contrast enhancement has been controversial for gliomas. Besides, there is little study on the influence of enhancement pattern on recurrence and survival in LGGs. The present study found that patients with ring-like enhancement exhibited significantly longer PFS time in the Kaplan–Meier survival curves. Consistent with previous studies [19], we observed other enhancement patterns (focal enhancement and diffuse enhancement) had no influence on the prognosis of LGGs. None of these ten patients with ring-like enhancement had disease progression or died after surgery and chemoradiotherapy, hence we cannot use the Cox proportional hazards model to analyze the effect of ring-like enhancement on survival for the multivariate analysis. The contrast enhancement of gliomas mainly reflects the disruption of the blood–brain barrier (BBB), increasing or decreasing the abnormal permeability of BBB would influence the area and morphology of enhancement pattern [24]. The phenomenon of ring-like enhancement might be caused by peripheral displacement of vessels when the tumor enlarges. The ring-like pattern might affect the abnormal permeability thereby longer the PFS time in patients.

Necrosis is thought to be the most important pathological prognostic factor in gliomas [25]. Several groups have shown that the extent of necrosis is correlated significantly with poor survival in glioblastoma [23,26]. Some authors reported that necrosis was the best predictor as an MRI variable in grading gliomas [27]. However, few attempts have been made to explore the prognostic significance of tumor necrosis in LGGs. In the present study, there was no significant difference in PFS and OS between patients who had LGGs with necrosis and those with no necrosis. Perhaps because the deficient number of cases with necrosis impacts the result of the present study, or maybe the mechanism of necrosis in LGGs is different from the high grade.

After multivariate analyses of all unfavorable prognostic factors and cysts formation, the diameter of tumor (≥6 cm) retained significance as unfavorable prognostic factors, just as the EORTC study 22844 pointed out [10]. In addition, the results showed that cysts formation was an independent indicator of favorable prognosis. Previous studies have evaluated the association between cysts and prognosis in LGGs. Both studies suggested that the presence of cysts tended to have a better prognosis, but both did not reach statistical significance [17,28]. This study showed that the patients with a cystic component exhibited a significantly longer PFS time and that cysts were an independent prognosis factor. One proposed explanation is that the cyst formation may be related to slower tumor growth and a clear margin, hence tumors with cyst are less aggressive and have a better prognosis [28]. Another proposed mechanism to explain is that cysts formation implies more indolent neoplasm growth, which can increase survival [16].

The optimum treatment of LGGs remains controversial, particularly on the issues of radiotherapy dosage. Radiotherapy can cause adverse long-term effects such as late neurocognitive toxicity and leukoencephalopathy. The EORTC 22844 [29] and NCCTG [30] studies suggested that comparing with ‘low’ doses, radiotherapy with ‘high’ doses will not give the patients of LGGs a survival benefit (59.6 vs. 45 Gy and 64.8 vs. 50.4 Gy, respectively). In the present study, the results indicated that cysts formation and ring-like enhancement means better prognosis. Perhaps the conventional radiotherapy dosage for these patients is not required, which could be explored in the further study.

However, there are several limitations in the present study, First, it is better for the retrospective study to have greater sample size and a longer follow-up period so that we can fully explore the clinical prognosis significance of MRI features, however the statistical results of these existing cases are still precious as they pointed out the direction of future research and our group is still collecting and analyzing new LGGs samples in clinical work to improve our sample size and further validate the research conclusion. Moreover, the pathophysiology of ring-like enhancement and cyst formation remains unclear, future studies are needed to explore the mechanism to affect prognosis in LGGs.

## Conclusion

In this retrospective study, we analyzed the clinical data of 80 patients with LGGs (WHO grade II). The results showed that cyst formation on preoperative MR images is an independent indicator of favorable prognosis. In addition, tumor with ring-like enhancement pattern tends to have a longer survival. Our findings indicated that cysts and ring-like enhancement on routine preoperative MRI scans can be the reference marks in helping to predict the survival outcomes in patients with LGGs.

## Abbreviations

BBB: blood–brain barrier
EORTC: European Organisation for Research and Treatment of Cancer
HR: hazard ratio
IDH: Isocitrate dehydrogenase
KPS: Karnofsky Performance Status
LGG: low-grade glioma
MRI: magnetic resonance imaging
OS: overall survival
PFS: progression-free survival
T1-W: T1-weighted imaging
T2-W: T2-weighted imaging
WHO: World Health Organization
95%CI: 95% confidence interval
